The article "Multidrug-Resistance Related Long Non-Coding RNA Expression Profile Analysis of Gastric Cancer" was retracted in 2019. Reasons: duplicated images; unreliable results or conclusions.

# Multidrug-Resistance Related Long Non-Coding RNA Expression Profile Analysis of Gastric Cancer

**DOI:** 10.1371/journal.pone.0135461

**Published:** 2015-08-20

**Authors:** Ying Wang, Kaichun Wu, Zhiping Yang, Qingchuan Zhao, Dongmei Fan, Po Xu, Yongzhan Nie, Daiming Fan

**Affiliations:** 1 State Key Laboratory of Cancer Biology and Xijing Hospital of Digestive Diseases, Fourth Military Medical University, 15 Changlexi Road, Xi’an, Shaanxi, China; 2 Department of Oncology, First Affiliated Hospital of Henan University of Science and Technology, 24 Jinghua Road, Luoyang, Henan, China; 3 Department of Gynaecology and Obstetrics, First Affiliated Hospital of Henan University of Science and Technology, 24 Jinghua Road, Luoyang, Henan, China; 4 Department of Urology, First Affiliated Hospital of Henan University of Science and Technology, 24 Jinghua Road, Luoyang, Henan, China; H.Lee Moffitt Cancer Center & Research Institute, UNITED STATES

## Abstract

The effect of chemotherapy of gastric cancer (GC) remains very poor because of multidrug resistance (MDR). However, the mechanisms underlying MDR of GC remains far from fully understood. The aim of this study is to illustrate the potential mechanisms of the MDR of GC at mainly the long non-coding RNA (lncRNA) level. In this study, GC cell line, SGC7901, and two MDR sublines, SGC7901/VCR and SGC7901/ADR were subjected to an lncRNA microarray analysis. Bioinformatics and verification experiments were performed to investigate the potential lncRNAs involved in the development of MDR. Pathway analysis indicated that 15 pathways corresponded to down-regulated transcripts and that 20 pathways corresponded to up-regulated transcripts (p-value cut-off is 0.05). GO analysis showed that the highest enriched GOs targeted by up-regulated transcripts were “system development” and the highest esenriched GOs targeted by the down-regulated transcripts were “sterol biosynthetic process”. Our study is the first to interrogate differentially expressed lncRNAs in human GC cell line and MDR sublines and indicates that lncRNAs are worthwhile for further study to be the novel candidate biomarkers for the clinical diagnosis of MDR and potential targets for further therapy.

## Introduction

Multidrug resistance (MDR) remains a major obstacle for chemotherapy failure in the treatment of gastric cancer, which is a leading cause of cancer-related death worldwide. Multiple multidrug resistance-associated proteins (MRPs)[1] or miRNAs[2] that mediate MDR through different mechanisms have been previously identified. However, the mechanisms underlying MDR of GC remains far from fully clear.

Genomes sequencing indicated that eukaryote genomes encode a surprisingly large number of noncoding transcripts compared with prokaryote genomes. Among these noncoding transcripts, many are long non-coding RNAs (lncRNAs) which play important roles in regulating mRNA transcription or translation at transcriptional or post-transcriptional levels. lncRNAs are RNAs that lack coding potential, which are >200 bp and account for at least 80% of the transcripts of the entire genome[3]. Accumulating data indicate that lncRNA plays important roles in the regulation of mRNA[4], organelle biogenesis[5], the subcellular trafficking of molecules[6], and cell development [7] [8].

The article "Multidrug-Resistance Related Long Non-Coding RNA Expression Profile Analysis of Gastric Cancer" was retracted in 2019. Reasons: duplicated images; unreliable results or conclusions.

LncRNA dysregulation was involved in multiple types of diseases, including cancer^[^ ^4^ ^,^ ^9^ ^,^ ^10^ ^]^. Namely, lncRNAs may play important roles in the carcinogenesis, metastasis and invasiveness of multiple malignant tumors through affecting oncogene expression. For example, the COX-2-lncRNA, PACER, may act as a new potential target for COX-2-modulation in inflammation and cancer[11]; RNAi-mediated knock-down of LINC01081 in normal fetal lung fibroblasts showed that this lncRNA positively regulates FOXF1 transcript level, further indicating that decrease in LINC01081 expression can contribute to development of alveolar capillary dysplasia with misalignment of pulmonary veins[12]; lncRNA HOTAIR may also be a valuable predictor for colon cancer management[13] and MALAT1 might be considered as a potential prognostic indicator and may be a target for diagnosis and gene therapy for pancreatic duct adenocarcinoma [14]; overexpression of lncRNA H19 enhances carcinogenesis and metastasis of gastric cancer and the effect of H19 in GC is mediated by the direct upregulation of ISM1 and the indirect suppression of CALN1 expression via miR-675[15]. Hence, to get preliminary insight of the molecular mechanisms of MDR of GC, we studied the lncRNA expression profile of GC MDR sublines.

Here, we studied the differentially expression profiles of lncRNAs and mRNAs between GC cellline SGC7901 and MDR sublines SGC7901/ADR and SGC7901/VCR using lncRNA microarray analysis. Comparison of differentially expressed transcripts between the sublines and parental cellline revealed 15 pathways that corresponded to down-regulated transcripts and 20 pathways that corresponded to up-regulated transcripts (p value cut-off was 0.05). Gene ontology (GO) analysis showed that the most highly enriched GO terms for the up-regulated transcripts were “system development”, “nucleosome”, and “binding” and the most highly enriched GO terms for the down-regulated transcripts were “sterol biosynthetic process”, “cell periphery”, and “steroid dehydrogenase activity”. Our results showed that the lncRNA and mRNA expression profiles differed significantly between MDR sublines and parental celline. This finding suggests that the aberrant expression levels of lncRNAs might contribute to the development of MDR of GC. Further study of the differences in lncRNA expression profiles may provide new potential methods for reversing MDR phenotype of GC.

The article "Multidrug-Resistance Related Long Non-Coding RNA Expression Profile Analysis of Gastric Cancer" was retracted in 2019. Reasons: duplicated images; unreliable results or conclusions.

## Results

### Differentially expressed lncRNAs

The highthroghput lncRNA microarray data showed a total of 27,883 lncRNAs expressed in gastric cancer cellline, SGC7901 and two multidrug-resistance sublines, SGC7901/ADR and SGC7901/VCR(S1 Table). To infer the relationships among specimens, hierarchical clustering analysis was used to arrange celllines into groups according to their expression levels, presenting the relationships of the lncRNA expression modes between celllines (Fig 1A and 1B). Further study of these data exhibited an average of 1637 differentially expressed lncRNA. Among them, 638 were consistently up-regulated and 999 were consistently down-regulated (fold change≥2.0) (S2 Table). ASHG19A3A028863 (fold change:146.0139) was the most up-regulated lncRNA, and ASHG19A3A007184 (fold change:58.7105) was the most down-regulated lncRNA. Furthermore, down-regulated lncRNAs were more common than up-regulated lncRNAs in our microarray data(S2 Table).

**Fig 1:** Microarray analysis of MDR-related lncRNA of gastric cancer cell lines. A. The scatterplot of lncRNA expression profile. B. Heat map and hierarchical clustering dendrogram of lncRNA chips.

### Differentially expressed mRNAs

There were 19,644 mRNAs identified in the GC MDR sublines analyzed by mRNA expression profiling data using microarray analysis and the Hierarchical clustering analysis presented the relationships among the mRNA expression modes that were present in the GC MDR sublines and their parental celline (Fig 2A and 2B) (S3 Table). Among the differentially expressed mRNA between SGC7901/ADR, SGC7901/VCR and SGC7901, 730 was consistently up-regulated and 650 was consistently down-regulated in SGC7901/ADR and SGC7901/VCR celllines compared with SGC7901 (Fig 2B). (S4 Table). NM_000735 (gene symbol: CGA, fold change: 106.19) was the most up-regulated mRNA, and NM_001136574 (gene symbol: LANCL1, fold change: 25.43) was the most down-regulated mRNA (Fig 2B).

**Fig 2:** Microarray analysis of MDR-related mRNA of gastric cancer cell lines. A. Heat map and hierarchical clustering dendrogram of mRNA chips. B. Forms showing top 10 differentially expressed mRNAs.

### GO analysis

To determine the gene and gene product attributes in biological processes, cellular components and molecular functions, Gene Ontology (GO) analysis was performed hereby. Fisher’s exact test is done to test if there is more overlap between the DE list and the GO annotation list than would be expected by chance. The p-value denotes the significance of GO terms enrichment in the DE genes. The lower the p-value, the more significant the GO Term (p-value< = 0.05 is recommended). It showed that the highest enriched GOs targeted by up-regulated transcripts were tissue homeostasis (GO:0048731; ontology: biological process; p = 6.84E-08) (Fig 3A), nucleosome (GO:0000786; ontology: cellular component; p = 2.10E-07) (Fig 3B) and binding (GO:0005488; ontology: molecular function; p = 0.001) (Fig 3C) and that the highest enriched GOs targeted by the down-regulated transcripts were sterol biosynthetic process (GO:0016126; ontology: biological process; p = 0.000) (Fig 3D), cell periphery (GO:0071944; ontology: cellular component; p = 3.80E-06) (Fig 3E) steroid dehydrogenase activity (GO:0016229; ontology: molecular function; p = 0.001) (Fig 3F) (S5 Table).

The article "Multidrug-Resistance Related Long Non-Coding RNA Expression Profile Analysis of Gastric Cancer" was retracted in 2019. Reasons: duplicated images; unreliable results or conclusions.

**Fig 3:** Pie charts showing the significant enrichment terms. The pie chart shows the top ten counts of the significant enrichment terms. The ontology covers three domains: Biological Process, Cellular Component and Molecular Function. Fisher’s exact test is used to find if there is more overlap between the DE list and the GO annotation list than would be expected by chance. The p-value denotes the significance of GO terms enrichment in the DE genes. The lower the p-value, the more significant the GO Term (p-value< = 0.05 is recommended) (A-C) The highest enriched GOs targeted by up-regulated transcripts: A, Biological process (BP), B, Cellular component (CC), C, Molecular function (MF). (D-F) The highest enriched GOs targeted by down-regulated transcripts: A, Biological process (BP), B, Cellular component (CC), C, Molecular function (MF).

### Pathway analysis

In this study, pathway analysis exhibited that 20 pathways consistently corresponded to up-regulated transcripts and that the most enriched network was “Alcoholism—Homo sapiens (human)”(Fisher-P value = 3.66E-08) composed of 24 targeted genes (Fig 4A); furthermore, the pathway analysis also showed that 15 pathways consistently corresponded to down-regulated transcripts and that the most enriched network was “Steroid biosynthesis—Homo sapiens (human)”(Fisher-P value = 0.00044) composed of 5 targeted genes (Fig 4B) (S6 Table, the recommend p-value cut-off is 0.05). Among these pathways, the gene category “Circadian rhythm” disruption has been reported to be associated with various cancers, including gastric cancer[16], chronic myeloid leukemia[17], head and neck squamous cell carcinoma[18], hepatocellular carcinoma[19], endometrial carcinoma[20], and breast cancer[21]. The gene category“NOD-like receptor signaling pathway”, which consists of NOD1, has been showed that NOD1/CARD4 and NOD2/CARD15 gene polymorphisms may be associated with altered risk of gastric[22], colorectal[23], lung[24], laryngeal[25], gallbladder[26], pancreatic[27], small bowel, kidney[28], urinary bladder cancer[29], skin cancer, lymphoma[30] and leukemia[31]. Here, we further examined the expression and function of ARNT (aryl hydrocarbon receptor nuclear translocator) mediated MDR1(multidrug resistance 1) up-regulation pathway. It was found that ARNT and MDR1 were significantly up-regulated in SGC7901/ADR and SGC7901/VCR cell lines compared to SGC7901, the effect of significant up-regulation of MDR1 mediated by ARNT expression vector transfection was compromised via Sp1 siRNAs transfection. Plate colony formation assay showed that SGC7901/ADR cell colony formation rates were remarably higher in pARNT+/siSp1- group compared with pARNT+/siSp1+ group with the adriamycin(ADR) supplement into the culture meida (p < 0.0001) (Fig 5).

The article "Multidrug-Resistance Related Long Non-Coding RNA Expression Profile Analysis of Gastric Cancer" was retracted in 2019. Reasons: duplicated images; unreliable results or conclusions.

**Fig 4:** Representational pathway schematic diagrams. (A) Pathway: Alcoholism—Homo sapiens (human). (B) Pathway: Steroid biosynthesis—Homo sapiens (human).The bar plot shows the top ten Enrichment score (-log10 (P value)) value of the significant enrichment pathway. Yellow marked nodes are associated with down-regulated genes, orange marked nodes are associated with up-regulated or only whole dataset genes, green nodes have no significance.

**Fig 5:** ARNT–MDR1 pathway mediated the drug-resistance phenotype gastric cancer. (A) expression of ARNT, MDR1 and Sp1, a, western blotting, b, qRT-PCR. (B) The effect of siARNT transfection on the expression of ARNT, MDR1 and Sp1, a, western blotting, b, qRT-PCR of SGC7901/ADR, c, qRT-PCR of SGC7901/VCR. (C) The effect of pARNT (ARNT expression vector) and siSp1 transfection on the expression of ARNT, MDR1 and Sp1, a, western blotting, b, qRT-PCR of SGC7901/ADR. (D) Plate colony formation assay of SGC7901/ADR cells with the adriamycin supplement into the culture media (1μg/ml) at the designated time. (Data were means of three separate experiments (mean ± SEM), one-way ANOVA analysis, *** p < 0.0001).

### Real time quantitative PCR validation

To examine the microarray data, six up-regulated lncRNAs and ten under-regulated lncRNAs were randomly selected from the consistently differentially expressed lncRNAs using SGC7901/ADR, SGC7901/VCR and SGC7901 cellines and the qRT-PCR results and microarray data are consistent(Fig 6A); to further study the expression levels of the these lncRNAs in drug-resistant gastric tissues, twenty drug-resistant gastric samples and paired non multidrug-resistant tissues were examined for the expression level of these lncRNAs using quantitative real-time PCR (qRT-PCR) (Fig 6B).The results demonstrated that gastric cancer samples treated with ADR for 5 days exhibited significant difference of expression levels of these sixteen lncRNAs afformentioned compared with control groups(Fig 6C). Moreover, correlation analysis showed that lncRNA NR_015379 expression levels were negatively correlated with the inhibition rates of these twenty drug-resistant gastric samples (Fig 6D and 6E, p < 0.01).

The article "Multidrug-Resistance Related Long Non-Coding RNA Expression Profile Analysis of Gastric Cancer" was retracted in 2019. Reasons: duplicated images; unreliable results or conclusions.

**Fig 6:** LncRNA chosen randomly for examination using qRT-PCR assay. (A) Sixteen lncRNAs expression levels in SGC7901/ADR and SGC7901/VCR celllines compared with SGC7901 celline. (B) Schematic diagram of gastric cancer samples treated with HDRA followed by qRT-PCR and inhibition rate assay.(C) Sixteen lncRNAs expression levels in twenty gastric cancer samples treated with ADR compared with control groups.(D-E) lncRNA NR_015379 expression levels were negatively correlated with the inhibition rates of gastric cancer samples treated with ADR.

## Discussion

Our previous research has already found that miR-21 may promote the drug resistance of various cancers[32]; LncRNA-MRUL promotes ABCB1 expression in multidrug-resistant gastric cancer cell sublines[33]; CUTL1 activity is inversely associated with drug resistance and thus is an attractive therapeutic target to modulate multidrug resistance in gastric cancer[34]; gastric CSCs were identified from VCR-preconditioned SGC7901 cell line, characterized by high tumorigenicity and the capacity for self-renewal and differentiation[35]; MAD2 might play an important role in the development of human gastric cancer and that silencing the MAD2 gene may help to deal with the multidrug resistance of gastric cancer cells[36] and hypoxia-elicited MGr1-Ag/37LRP expression activated by HIF-1 depends on ERK activation. These events are dependent of reactive oxygen intermediates[37].However, the multidrug resistance mechanisms of GC are far more elucidated and lncRNAs dysregulation of GC MDR sublines have not been studied yet.

In this study, GC cell line, SGC7901, and two MDR sublines, SGC7901/VCR and SGC7901/ADR were subjected to an lncRNA microarray analysis. Bioinformatics and verification experiments were performed to investigate the potential lncRNAs involved in the development of MDR. Pathway analysis indicated that 15 pathways corresponded to down-regulated transcripts and that 20 pathways corresponded to up-regulated transcripts (p-value cut-off is 0.05). GO analysis showed that the highest enriched GOs targeted by up-regulated transcripts were “system development” and the highest esenriched GOs targeted by the down-regulated transcripts were “sterol biosynthetic process”.

The article "Multidrug-Resistance Related Long Non-Coding RNA Expression Profile Analysis of Gastric Cancer" was retracted in 2019. Reasons: duplicated images; unreliable results or conclusions.

Increasing evidence showed that lncRNA (long non-coding RNA) could play important roles in carcinogenesis and tumor invasion and metastasis[38]. For example, John[39] etc demonstrated that lncRNA *PCGEM1* is associated with prostate cancer; transforming growth factor-β-induced lncRNA-Smad7 was found to inhibit apoptosis of mouse breast cancer JygMC (A) cells and thus suggest ed a complex mechanism for regulating the anti-apoptotic and tumor-progressive aspects of TGF-β signaling[40]; lncRNA, prostate cancer–associated transcript 29 (PCAT29), was characterized along with its relationship to the androgen receptor, functioned as an androgen-regulated tumor suppressor in prostate cancer[41]; Yuan etc discovered a novel TGF-β-induced lncRNA, lncRNA-ATB, which stimulated EMT through sequestering miR-200s and facilitated colonization by stabilizing *IL-11* mRNA, thus promoting both early and late steps of cancer metastasis[42].

It has been found that lncRNAs play pivotal roles in altering the expression of protein-coding genes via cis- or trans-mechanisms. Here we found that lncRNAs up-regulated in SGC7901/ADR and SGC7901/VCR compared with SGC7901lncRNA such as AF119893,which was intronic antisense to NRP2 (Neuropilin-2). It has been suggested that the NRP2/VEGF-C axis plays a role in bladder cancer therapy resistance and the VEGF-paxillin-NRP2 pathway could represent a new therapeutic target for cancer and other angiogenesis-related diseases. lncRNA AF461897 was intron sense-overlapping of ABCB9. Dong etc has demonstrated that miR-31 exerted an anti-apoptotic effect most likely through the inhibition of ABCB9 and thus provide a novel strategy involving the use of miR-31 as a potential target in NSCLC chemotherapy. lncRNA BC065904 was intron sense-overlapping of CTBP2, one of the transcriptional corepressors of C-terminal binding protein (CtBP) family, which functioned as a corepressor of E2F7 and as a regulator of DNA damage response. lncRNA NR_026900 was exon sense-overlapping of QSOX1, which was demonstrated to reduce proliferation, migration and invasion of breast cancer cells in vitro and reduces tumor growth in vivo.

On the other hand, lncRNAs down-regulated in SGC7901/ADR and SGC7901/VCR compared with SGC7901lncRNA such as AF113689 was natural antisense to RRM1. Khatri etc have reported that pre-exposure of RRM1 siRNA decreased the IC50 value of Gemcitabine hydrochloride 5 folds in A-549 cells compared to Gemcitabine hydrochloride alone, indicating that RRM1 was a potential oncogene of lung cancer. lncRNA uc010iyh was intronic antisense of NAIP (Neuronal Apoptosis Inhibitory Protein), which is one of the IAP-family. It has been shown that IAPs could be involved in prostate disorder (BPH, PIN and PC) development since might be provoke inhibition of apoptosis and subsequently cell proliferation. LncRNA uc003jsd was exon sense-overlapping of PDE4D,i.e, cAMP-specific 3',5'-cyclic phosphodiesterase 4D. Lin etc showed that PDE4D functions as a tumor-promoting factor and represents a unique targetable enzyme of cancer cells. LncRNA NR_002332 was exon sense-overlapping of ST7, suppressor of tumorigenicity 7, which has been proposed to be a tumor suppressor gene in the chromosome region 7q31.1-q31.2.

The article "Multidrug-Resistance Related Long Non-Coding RNA Expression Profile Analysis of Gastric Cancer" was retracted in 2019. Reasons: duplicated images; unreliable results or conclusions.

Pathway analysis revealed potential pathways involved in the development of multidrug resistance (MDR) of gastric cancer. ARNT was one of the 20 pathways consistently corresponded to up-regulated transcripts and was reported to be involved in the multidrug resistance development of multiple malignant tumors[43], including multiple myeloma[44], and AML (acute myeloid leukemia)[45]. MDR1 encodes P-glycoprotein which is an energy-dependent efflux pump that could export planar hydrophobic molecules including some chemotherapeutic drugs such as adriamycin, cisplatin, taxol and so on from the cell[46, 47]. Here, we found that ARNT and MDR1 were significantly up-regulated in SGC7901/ADR and SGC7901/VCR cell lines compacared to SGC7901, the effect of significant up-regulation of MDR1 mediated by ARNT expression vector transfection was compromised via Sp1 siRNAs transfection, which indicated the role of ARNT-MDR1pathway in the MDR phenotype of gastric cancer.

Further investigation showed that some protein-coding genes involved in the drug-resistance phenotype and development of malignant tumors maybe were cis-regulated by correlated lncRNAs. For example, ABCB1(ATP-binding cassette, sub-family B (MDR/TAP), member 1, P-glycoprotein(P-gp) coding gene), located 400Kb upstream of lncRNA MRUL (NR_024549: MDR-related and up-regulated lncRNA), was significantly up-regulated through a potential enhancement-like role played by MRUL and promoted drug-resistance phenotype of SGC7901/ADR and SGC7901/VCR cells[33]; ADAM22, a candidate gene for malignant transformation of ovarian endometriosis[48], was correlated with lncRNA AL133090 in a exon sense-overlapping way; PLCG1 was correlated with lncRNA AK021471 in a intron sense-overlapping way and recurrent mutations in PLCG1 was identified in angiosarcomas[49]; FYN was correlated with lncRNA AK AK090692 in a intron sense-overlapping way and antagomir-1290 suppresses CD133(+) cells in non-small cell lung cancer by targeting fyn-related Src family tyrosine kinase[50], etc.

The article "Multidrug-Resistance Related Long Non-Coding RNA Expression Profile Analysis of Gastric Cancer" was retracted in 2019. Reasons: duplicated images; unreliable results or conclusions.

This study demonstrated that deregulation of lncRNAs was involved with the development of multidrug-resistance phynotype of gastric cancer. Further analysis of these lncRNAs and related pathways could provide insight to the mechanisms of chemotherapy drug resistance of gastric cancer and provide novel directions for reverse multidrug resistance phynotype.

## Materials and Methods

### Ethics statement

All of the experimental procedures were approved by the Institutional Review Board of the Fourth Military Medical University. Written informed consent was obtained for all patient samples.

### Cell lines and cell culture

The human GC cell line SGC7901 was obtained from the Academy of Military Medical Science (Beijing, China). Two multidrug-resistant sublines, SGC7901/VCR and SGC7901/ADR, were developed in our lab [51]. SGC7901/VCR, SGC7901/ADR and SGC7901 were grown in RPMI1640 medium (Thermo Scientific Co., USA) that was supplemented with 10% fetal calf serum (FCS) (Thermo scientific Co., USA) in a humidified incubator with 5% CO2 at 37°C. VCR (1.0 μg/ml) or ADR (0.5 μg/ml) was added into the culture medium of the appropriate cells to maintain the drug-resistant phenotype.

### RNA isolation, labeling and array hybridization

Total RNA was harvested from SGC7901, SGC7901/ADR and SGC7901/VCR using TRIzol reagent (Invitrogen, CA, USA) and the RNeasy Kit(Qiagen Co.,Germany) according to manufacturer's instructions, including a DNase digestion step. Total RNA from each cellline was quantified using a NanoDrop ND-1000(OD 260 nm, NanoDrop,Wilmington, DE), RNA integrity was assessed using standard denaturing agarose gel electrophoresis, and the purity was judged by the ratio of absorbance at 260 nm to 280 nm (A260/A280). Double-strand cDNA (ds-cDNA) was synthesized using 5 μg total RNA by an Invitrogen SuperScript ds-cDNA synthesis kit in the presence of 100 pmol oligo dT primers. Then, the ds-cDNA was labeled and performed hybridization as previously described[52]. The RNA labeling and microarray hybridization was performed by KangChen Bio-tech, Shanghai, PR China.

### Highthroughput lncRNA expression profile analysis

Qualified RNA was used to synthesize double-stranded cDNA using Superscript Double-Stranded cDNA Synthesis Kit(Invitrogen Co., USA). Double-stranded cDNA was labeled and hybridized to the human LncRNA microarray V2.0(Arraystar Co. USA). microarray V2.0 contains about 33,000 lncRNAs collected from the authoritative data sources including NCBI RefSeq, UCSC, RNAdb, LncRNAs from literatures and UCRs. Sequences were selected with proprietary strategies. Repeat sequences and ncRNAs shorter than 200 bp were deleted. To enhance statistical confidence, each human lncRNA array was composed of 60,302 distinct probes (60 mers) and each transcript was represented by 1–5 probes. Each transcript was represented by a specific exon or splice junction probe to identify individual transcripts accurately. The microarray hibridization and bioinformatic analysis was performed by KangChen Bio-tech, Shanghai, PR China. The raw intensity data and normalized data were shown in Gene Expression Omnibus (GSE69342: http://www.ncbi.nlm.nih.gov/geo/query/acc.cgi?acc=GSE69342).

The article "Multidrug-Resistance Related Long Non-Coding RNA Expression Profile Analysis of Gastric Cancer" was retracted in 2019. Reasons: duplicated images; unreliable results or conclusions.

### Quantitative real-time PCR (qRT-PCR)

The total RNA of SGC7901, SGC7901/ADR and SGC7901/VCR was isolated using TRIzol reagent (Invitrogen,CA, USA) and was then reverse transcribed using PrimeScript RT reagent Kit with gDNA Eraser (Perfect Real Time) (TaKaRa, Dalian China) according to the manufacturer’s structions. The expression of eight up-regulated lncRNAs and six down-regulated lncRNAs was measured by qRT-PCR using SYBRGreen assays (TaKaRa, Dalian, China), and GAPDH was used as an internal control. The primers are listed in Table 1. The expression level of each lncRNA was represented as fold change using 2-△△Ct methods. The expression level of lncRNAs differentially expressed between SGC7901 and MDR sublines SGC7901/ADR and SGC7901/VCR were analyzed using Student’s t-test with SPSS (Version 17.0 SPSS Lnc). A value of p < 0.05 was considered significant.

**Table 1:** Primers used for qRT-PCR.

Name	regulated	Forward (5’→3’)	Reverse (5’→3’)	Tm (°C)	Length (bp)
NR_024596	up	TCCTAGAGATGGGAGGATGCC	TCCAAAAGAGAGGGTTCTGTGCT	60	130
NR_024421	up	TGCCGCCTTCCAATCAAATG	TCTCGTCCTCCCAGCGAAAT	60	175
NR_024606	up	CGTGGGGAATGGACCCATAG	GGACTTGCCCTTGGTGACTC	60	197
NR_003595	up	AGGACCCCCTGACAGATAGC	AGCTTCTTAGGTGGAAAGCAA	60	183
NR_015379	up	ACGCTAACTGGCACCTTGTT	CCGGACTGCTTCAAGTGTGA	60	122
NR_015381	up	GAGCTGTCCTAACTCTGCGG	GAGGGTTGGGTACCTTCGTG	60	123
NR_024510	down	GCGTTGATTTCTTGGCACCC	GGTTCACAACTCCCCTGCTT	60	173
NR_002763	down	TAGGCCTAGGAGCTAGCGAT	ACAAAGGGAGTGCGGTACAT	60	103
NR_002712	down	TGTCTGGGTTTGTGGAACCT	GCAGAACAGCATGATCGCAG	60	194
NR_015360	down	TGGCTGATAGCTCATTGCCC	GGCCCTTTGGTAGCAAACAC	60	212
NR_002768	down	GTAGGTGTTTGGGTGCTCGC	GAATCGGGTCTGTGGACCTC	60	280
NR_026860	down	GGGAGCTTGAGCTGAGATGG	TCTTCTCGCAAAAGGCGAGT	60	125
Name	regulated	Forward (5’→3’)	Reverse (5’→3’)	Tm (°C)	Length (bp)
NR_024596	up	TCCTAGAGATGGGAGGATGCC	TCCAAAAGAGAGGGTTCTGTGCT	60	130
NR_024421	up	TGCCGCCTTCCAATCAAATG	TCTCGTCCTCCCAGCGAAAT	60	175
NR_024606	up	CGTGGGGAATGGACCCATAG	GGACTTGCCCTTGGTGACTC	60	197
NR_003595	up	AGGACCCCCTGACAGATAGC	AGCTTCTTAGGTGGAAAGCAA	60	183
NR_015379	up	ACGCTAACTGGCACCTTGTT	CCGGACTGCTTCAAGTGTGA	60	122
NR_024433	down	AGCATCCACGTTGTATCCCC	CCTGCTCCCTCTCCGTAAAC	60	183
NR_027267	down	AATGCTGGACCAGATGACCC	TACCCAAAGACATTCCACGGG	60	142
ARNT	up	TACCCGCTCAGGCTTTTCTG	CTGCTGTCCGTGTCTGGAAT	60	236
MDR1	up	GGAAAGTGCTGCTTGATGGC	AGGCATGTATGTTGGCCTCC	60	195
Sp1	down	CAGGACCCCCTTGAGCTTGTC	CCTGTTCCCCCTGACTGACT	60	307

Histoculture Drug Response Assay (HDRA) Fresh GC tumor tissue was harvested from each surgically resected specimen and placed in a 24-well plate. Cubes of collagen gel sponge(1 cm^3^) were immersed in 1 mL RPMI 1640 supplementing with 20% fetal bovine serum. Tumor tissues were placed onto collagen sponge following ADR were added at a final concentration of 6 μg/mL and they were incubated at 37°C with 5% CO2. Tumor tissues treated with normal saline (N.S) without ADR were used as control. Evaluation and calculation methods are as previously described[53]. The inhibition rate (IR) of tumor growth = (1-mean absorbance of treated wells per gram of tumor/mean absorbance of control wells per gram of tumor) ×100. In this study, the IR cut-off value equal to or greater than 30% (IR30) was defined as chemosensitivity according to preliminary study result[54]. Just as instructed, the clinic pathological information of the tumor tissue’s source used for HDRA should be given respectively were presented in Table 2.

The article "Multidrug-Resistance Related Long Non-Coding RNA Expression Profile Analysis of Gastric Cancer" was retracted in 2019. Reasons: duplicated images; unreliable results or conclusions.

**Table 2:** Clinicopathologic characteristics for 20 patients with gastric cancer.

Characteristics	N	%
Age(years)		
>50	13	65
≤50	7	35
Histologic grade		
I	2	10
II	12	60
III	6	30
Lymphmatic metastasis		
Yes	14	70
No	6	30
TNM stage		
I	1	5
II	7	35
III/IV	12	60
Tumor size(cm)		
>5	13	65
≤5	7	35

### Cell lines and culture conditions

The human GC cell line SGC7901 was obtained from the Academy of Military Medical Sciences (Beijing, China). Multidrug-resistant sublines SGC7901/VCR and SGC7901/ADR were developed in our lab. SGC7901/VCR, SGC7901/ADR, and SGC7901 were cultured in RPMI 1640 medium (Thermo Scientific, USA) supplemented with 10% fetal calf serum (FCS) (ThermoScientific) in a 5% CO2 humidified incubator at 37°C. Vincristine (VCR;Sigma, Inc., St. Louis, MO; 1.0 μg/ml) and ADR (Sigma, Inc., St. Louis,MO; 0.5 μg/ml) were added to the culture medium of appropriate cell sublines to maintain the drug-resistant phenotype.

### Construction of pcDNA3.1(+)-ARNT plasmid

To over-express ARNT, pcDNA3.1(+)-ARNT plasmid was constructed. The human ARNT cDNA expression vector (pcDNA3.1(+)-ARNT) was constructed by CW Biotech Co. Ltd, Beijing, China. Briefly, the plasmid pcDNA3.1(+)-ARNT was generated according to the cDNA sequence from GenBank. The ARNT gene was generated by PCR amplification. The plasmid pcDNA3.1(+) was extracted through a Maxi Preparation kit (Omega, Georgia, USA). The PCR product was subcloned into the BamHI (Takara, Mountain View, USA) and HindIII (Takara) sites of pcDNA3.1 plasmid by T4 ligase (Takara, Mountain View, USA). The pcDNA3.1(+)-ARNT construct was verified by DNA sequencing (Invitrogen, Grand Island, USA) (data not shown).

The article "Multidrug-Resistance Related Long Non-Coding RNA Expression Profile Analysis of Gastric Cancer" was retracted in 2019. Reasons: duplicated images; unreliable results or conclusions.

### Generation of ARNT stable cell lines

SGC7901/ADR cell were cultured in 12-well plates with 1.0×10^5^ cells in each well, in an incubator with constant supply of 5% CO2 at 37°C. The medium was changed 24 h later with different concentrations of G418 antibiotic G418 (600 μg/mL) and replaced every 3 days for 14 days after cell culture. Parental cells were transfected with the pcDNA3.1(+)-ARNT plasmids using Lipofectamine 2000 according to the manufacturer’s instructions. The density of cells was 2×10^5^ cells per well in six-well plates. Monoclonal cell colony with G418 resistance was generated using the limiting dilution method by culturing single cell in 100 μL medium in 96-well plates for 24 h. Monoclonal cell colonies were digested 15 days later for further amplification to culture cells with stable ARNT expression in 24-well plates. Cells were transferred to cell culture flask until there was approximately 90% confluent. The ARNT over-expressed cell lines transfected by pcDNA3.1(+)-ARNT were named as SGC7901/ADR ARNT.

### Small interference RNA (siRNA) transfection

To knockdown the ARNT mRNA expression, siRNA transfection was performed. For transfections, Lipofectamine 2000 (Invitrogen, Carlsbad, CA, USA) and 50 nM siRNA (Gene Pharma Co., Shanghai, China) were used according to the manufacturer’s recommendations as described previously [55]. The siRNA sequences used are: 5′-AGUUUAUCCACAUCAUCUGGG-3′,5′-CAGAUGAUGUGGAUAAACUUC-3′.

### Western blotting

Total cell protein were lysed using lysis buffer supplemented with phenylmethylsulfonyl fluoride (1mM) on ice. Then, protein was electrophoresed through 12% SDS polyacrylamide gels and transferred to a PVDF membrane (Millipore, Massachusetts, USA). 5% non-fat milk powder was used to block membranes at room temperature for 1 h and the primary antibodies were incubated overnight. Next, membranes were incubated with secondary antibodies labeled with HRP for 1 h at room temperature after three 10-min washes in triethanolamine buffered saline solution with Tween (TBS-T). Finally, the signals were detected using an ECL kit (Pierce Biotech., Rockford, IL, USA) and the membranes were scanned and analyzed using a ChemiDoc XRS+ (Bio-Rad, California, USA) imaging system with imaging software (Version 1.0). Tubulin was used as an internal control. The Spectra multicolor broad-range protein ladder (Beyotime, Jiangsu, China) was used as a molecular marker. The antibodies used in the western blotting assay can be seen in the Table 3.

The article "Multidrug-Resistance Related Long Non-Coding RNA Expression Profile Analysis of Gastric Cancer" was retracted in 2019. Reasons: duplicated images; unreliable results or conclusions.

**Table 3:** Antibodies used in western blotting assay.

Antibody name	Producer/product code	Molecular weight	Origin	dilution
ARNT	Cell signaling technology/3414	87 kDa	Rabbit	1:1000
MDR1	Santa Cruz Biotechnology/ sc-55510	170kDa	Mouse	1:500
Sp1	Abcam/ab51513	81kDa	Mouse	1:100
Tublin	Abcam/ab6046	50 kDa	Rabbit	1:500

### Plate colony formation assay

The log-phase cells were harvested, plated into six-well plates (1×10^4^ cells/well), and chemotherapeutic drugs were added into the culture medium on the second day. The resulting colonies were stained with Coomassie Brilliant Blue (Sigma, Inc., St. Louis, MO, USA), and the visible colonies were counted after 2 weeks.

### Data analysis

In this study, informatic data analysis were performed by KangChen Biotech(Shanghai, PR China).All of the slides were scanned at 5 lm/pixel resolution using an Axon GenePix 4000B scanner (Molecular Devices Corporation) runed by GenePix Pro 6.0 software (Axon). Scanned images (JPEG format) were then performed grid alignment and expression data analysis using NimbleScan software (version 2.5). Expression data were normalized through Robust Multichip Average (RMA) algorithm included in the NimbleScan software. Moreover, the probe level files and mRNA level files were generated following normalization. All gene level files were imported into Agilent GeneSpring GX software (version 11.5.1) and normalized by the quantile method; then, Combat software was used to adjust the normalized intensity to remove batch effects. Significantly differentially expressed lncRNAs and mRNAs were identified through Volcano Plot filtering. Hierarchical clustering was performed using Agilent GeneSpring GX software (version 11.5.1)[56]. Data were expressed as means ± standard deviation (SD). Linear correlation analysis was performed using Pearson method in SPSS, version 17.0 (SPSS Inc., Chicago, IL). Differences were considered significant at a P value of < 0.05.

## Supporting Information

S1 Table The lncRNA expression profiling data. (XLS)

S2 Table The consistently up-regulated and down-regulated lncRNAs between SGC7901/ADR, SGC7901/VCR and SGC7901. (XLS)

S3 Table The mRNA expression profiling data. (XLS)

S4 Table The consistently up-regulated and down-regulated mRNAs between SGC7901/ADR, SGC7901/VCR and SGC7901. (XLS)

S5 Table Gene Ontology (GO) analysis. (XLSX)

S6 Table Pathway analysis. (XLS)
